# Research on Human Erythrocyte's Threshold Free Energy for Hemolysis and Damage from Coupling Effect of Shear and Impact Based on Immersed Boundary-Lattice Boltzmann Method

**DOI:** 10.1155/2020/8874247

**Published:** 2020-11-01

**Authors:** Zhong Yun, Chuang Xiang, Liang Wang

**Affiliations:** School of Mechanical and Electrical Engineering, Central South University, Changsha 410083, China

## Abstract

Researches on the principle of human red blood cell's (RBC) injuring and judgment basis play an important role in decreasing the hemolysis in a blood pump. In the current study, the judgment of hemolysis in a blood pump study was through some experiment data and empirical formula. The paper forms a criterion of RBC's mechanical injury in the aspect of RBC's free energy. First, the paper introduces the nonlinear spring network model of RBC in the frame of immersed boundary-lattice Boltzmann method (IB-LBM). Then, the shape, free energy, and time needed for erythrocyte to be shorn in different shear flow and impacted in different impact flow are simulated. Combining existing research on RBC's threshold limit for hemolysis in shear and impact flow with this paper's, the RBC's free energy of the threshold limit for hemolysis is found to be 3.46 × 10^−15^ J. The threshold impact velocity of RBC for hemolysis is 8.68 m/s. The threshold value of RBC can be used for judgment of RBC's damage when the RBC is having a complicated flow of blood pumps such as coupling effect of shear and impact flow. According to the change law of RBC's free energy in the process of being shorn and impacted, this paper proposed a judging criterion for hemolysis when the RBC is under the coupling effect of shear and impact based on the increased free energy of RBC.

## 1. Introduction

A high-performance blood pump is of critical importance, because it can function as an artificial heart for a short or long time to maintain the body's blood circulation [1]. Normalized index of hemolysis (NIH), which is the height of free hemoglobin in the hematocrit of 100 L blood being pumped out by a blood pump in unit time, is the blood pump's most important performance index [2]. In natural blood, the hemoglobin is intracellular. However, the hemoglobin will be dissociative because the RBC will be damaged by shear, impact, turbulence, and other mechanical factors when it passes through the high-speed spiral flow field of the blood pump [3, 4].

Experimental methods had been used in some papers for the research of RBC's damage in the blood pump; for example, a study of the RBC's threshold limit for hemolysis in shear flow by exposing the blood in a given shear rate of flow is proposed [5, 6]. Based on these experimental data, some empirical formulas have been proposed for the calculation of the degree of RBC's injury when the RBC is exposed in different shear stresses and times [7–9]. The RBC's threshold limit for hemolysis in impact flow by dropping the blood from a given height to the glass plate was researched by Yun and Tan [10]. However, the experimental method cannot explain the criteria of RBC's injury.

The RBC was often been modeled as a capsule that consisted of a capsule membrane and cytoplasm. The Skalak model (SK), the zero-thickness (ZT) shell model, and the neo-Hookean (NH) model are widely used to describe the properties of the capsule membrane [11]. However, three models can only respond to elastically for all based on the elasticity. Moreover, the surface area and volume of capsule cannot be conserved when no restraints are imposed on in NH model and ZT model. In a recent research, the nonlinear spring model was used to simulate the capsule membrane's resisting area and volume change [12, 13]. Considering the biological cell membrane's viscoelastic characteristics, the worm-like chain (WLC) model which is based on the spring model can perform better simulations of the membrane [14, 15].

In the study of RBC's injury model, Yun [3] has built the model of RBC's mechanical damage and researched the principle of RBC's rupture because of being impacted, pressure, shear stress, and turbulence. There are also some studies on RBC's behavior in microchannel, tank-treading motion and large deformation, and so on. Omori et al. [16] numerically investigated the dynamics of an RBC in a thin microprobe by combining the immersed boundary method and the finite element method. Xu et al. [17] presented IB-LBM to research the RBC's deformation and aggregation in the blood flow. Li et al. [18] employed dissipative particle dynamics in the study on RBC's tank-treading motion and motion frequency.

The RBC will be damaged when the increased free energy of RBC can offset the energy needed for RBC to be broken. In order to form a criterion of RBC's mechanical injury from the aspect of RBC's free energy, this paper takes the following approaches. Firstly, a nonlinear WLC model of RBC was presented and so was the immersed boundary and lattice Boltzmann method (IB-LBM), based on which the motion of RBC in plasma was numerically simulated. Secondly, the free energy, shape, and other parameters of RBC in shear and impact flow are analyzed. Third, the free energy of RBC that changed in the coupling effect of different shear stresses and different impact velocities was researched. And then, by combining the existing research on the RBC's threshold limit for hemolysis in shear and impact flow with this paper's, we get the threshold of free energy for RBC's damage which can be used as criteria for RBC's damage. The method for judging RBC's damage in coupling effects of shear and impact was proposed too. The research of this paper can provide the study of hemolysis in the blood pump with basis and foundation.

## 2. Model and Method

### 2.1. RBC Model

The membrane of RBC was modeled as a series of nonlinear wormlike chains as shown in Figure 1. The length change of the chain, the angle change of adjacent chains, and the change of area surrounded by all the chains can represent any deformation of RBC. When the shape of RBC was deformed, the energy which is defined as free energy of RBC is stored in chains. Based on the free energy change, the governing equations of the RBC deformation are [19, 20]

(1) $$\begin{array}{c} E_{\text{L}}=\underset{i=1,\cdots ,n}{\sum }k_{\text{L}}\frac{3x_{i}^{2}-2x_{i}^{3}}{1-x_{i}}, \end{array}$$

(2) $$\begin{array}{c} E_{\text{B}}=\underset{i=1,\cdots ,n}{\sum }k_{\text{B}}\left[1-\cos\left(\theta_{i}-\theta_{i0}\right)\right], \end{array}$$

(3) $$\begin{array}{c} E_{\text{s}}=\frac{k_{\text{s}}}{2}\left(\frac{S-S_{0}}{S_{0}}\right), \end{array}$$

(4) $$\begin{array}{c} F_{i}=-\frac{\partial E}{\partial r_{i}}+\frac{K_{Pi}}{l_{i}^{2}}\frac{\partial l_{i}}{\partial r_{i}}. \end{array}$$

*E*_L_, *E*_B_, and *E*_S_ are stretched/compressed energy, bending energy and area energy, respectively. *E* is the sum of *E*_L_, *E*_B_, and *E*_S_. *k*_L_, *k*_B_, and *k*_S_ are the chain constant for the change in length, bending angle change, and area change, respectively. The elastic chain force acting on the *i*th membrane node is *F*_*i*_. The total number of the chain elements is *n*. *x*_*i*_ = *l*_*i*_/*l*_*i*max_, set to 2.2 for the model [14], *l*_*i*_ is the length of the *i*th chain, and *l*_*i*max_ is the maximum extension of the *i*th chain. *θ*_*i*_ and *θ*_*i*0_ are the changed angle and reference angle between two chain elements, respectively. *S*_0_ is the reference area of the RBC, and *S* is the changed area. The second term of Equation (4) expresses the repulsive force between the neighboring nodes, and *K*_p*i*_ is calculated by using [21]

(5) $$\begin{array}{c} K_{Pi}=\frac{k_{\text{L}}l_{i0}^{2}}{l_{i\max}}\frac{4x_{i0}^{3}-9x_{i0}^{2}+6x_{i0}}{{\left(1-x_{i0}\right)}^{2}}. \end{array}$$

Vicoelasticity is an important property of RBC; the chains' viscosity in the WLC model can be expressed by [14]

(6) $$\begin{array}{c} F_{ij}^{D}=-\gamma^{T}u_{ij}-\gamma^{C}\left(u_{ij}\cdot e_{ij}\right)e_{ij}. \end{array}$$

*F*_*ij*_^*D*^ is the force acting on the particle. *γ*^*T*^ and *γ*^*C*^ are the coefficients and can be calculated from membrane viscosity *η*_*m*_ = 0.022 Pa∙s. Adding Equation (6) to Equation (11), the membrane viscosity can be analyzed using an algorithm.

The parameters of the RBC model are shown in Table 1. The model of RBC was verified by comparing the simulation result of RBC being stretched and experiment results of RBC being stretched by optical tweezers in our previous work [19, 20].

### 2.2. IB-LBM Method

The deformation of RBC in different flow relates to fluid-structure interaction problem. IB-LBM is applied to solve the interaction between the membrane and flow. The membrane was discretized to Lagrangian points, and the flow field was discretized to Eulerian points. An external forcing term is needed in order to adopt an immersed boundary method in the LBM; in the paper, we choose explicit-type split-forcing single-relaxation-time lattice Boltzmann equation with a forcing term [22]:

(7) $$\begin{array}{c} f_{\alpha }\left(x+e_{\alpha }∆t,t+∆t\right)=f_{\alpha }\left(x,t\right)-\frac{1}{\tau }\left[f_{\alpha }\left(x,t\right)-f_{\alpha }^{\left(\text{eq}\right)}\left(x,t\right)\right]+F_{\alpha }\left(x,\text{t}\right). \end{array}$$

Δ*t* is the streaming time step, *t* is the time, and *τ* is the single relaxation parameter. *f*_*α*_ is the density distribution function of the Eulerian point **x** along the *α* direction and *f*_*α*_^(eq)^ is its corresponding equilibrium state:

(8) $$\begin{array}{c} f_{\alpha }^{\left(\text{eq}\right)}=w_{\alpha }\rho \left[1+\frac{3}{c^{2}}\left(e_{\alpha }\cdot u\right)+\frac{9}{2c^{4}}\left(e_{\alpha }\cdot u\right)-\frac{9}{2c^{2}}u^{2}\right]. \end{array}$$

The discrete force distribution function *F*_*α*_(**x**, *t*) is

(9) $$\begin{array}{c} F_{\alpha }\left(x,t\right)=\left(1-\frac{1}{2\tau }\right)w_{\alpha }\left[3\frac{e_{\alpha }-u\left(x,t\right)}{c^{2}}+9\frac{e_{\alpha }\cdot u\left(x,t\right)}{c^{4}}e_{\alpha }\right]\cdot F\left(x,\text{t}\right). \end{array}$$

The membrane of RBC, which is a physical boundary, was discretized to Lagrangian points. And then, the boundary force is transformed into the forcing term *f* [23]:

(10) $$\begin{array}{c} f\left(r,t\right)=\int_{\Gamma }F\left(s,t\right)\delta \left(r-X\left(s,t\right)\right)ds. \end{array}$$

**F** is the force term at the Lagrangian points **X**, and *δ*(**r** − **X** (*s*, *t*)) is a delta function. The forcing term in the LBM is distributed to the Eulerian points by using a Dirac delta function [24]:

(11) $$\begin{array}{c} F_{ij}=\underset{b}{\sum }F_{b}D\left(x_{ij}-x_{b}\right)h^{2}, \end{array}$$

where **F**_*ij*_ and **F**_*b*_ are the force at the Eulerian point *ij* and Lagrangian point *b*, respectively. **x**_*ij*_, with coordinates (*x*_*ij*_, *y*_*ij*_), is the location of the Eulerian point *ij*. **x**_*b*_, with the coordinates (*x*_*b*_, *y*_*b*_), is the location of the Lagrangian point *b*. *h* is the grid size of the Eulerian mesh. *D*(**x**_*ij*_ − **x**_*b*_) can be expressed by

(12) $$\begin{array}{c} D\left(x_{ij}-x_{b}\right)=\frac{1}{h^{2}}d_{h}\left(\frac{x_{ij}-x_{b}}{h}\right)d_{h}\left(\frac{y_{ij}-y_{b}}{h}\right). \end{array}$$

The delta function is

(13) $$\begin{array}{c} d_{h}\left(r\right)=\left\{\begin{array}{c} \frac{1}{4}\left[1+\cos\left(\frac{\pi r}{2}\right)\right],\;\left|r\right|\leq 2,\\ 0,\;\left|r\right|>2. \end{array}\right. \end{array}$$

The velocity interpolation for the nearby Eulerian points is used for the position update of the Lagrangian points according to

(14) $$\begin{array}{c} u_{b}=\underset{i,j}{\sum }u_{ij}D\left(x_{ij}-x_{b}\right)h^{2}. \end{array}$$

Here, **u**_*b*_ and **u**_*ij*_ represent the velocities of the Lagrangian point *b* and the Eulerian point *ij*, respectively.

### 2.3. The RBC in Shear and Impact Flow

Two parallel plates moving in the same velocity *u* but in the opposite direction generated the shear flow, and the RBC was placed in the center of the flow field. In the Couette flow, when the distance between the two plates is *δ* (20 *μ*m in the paper), the kinetic viscosity of the fluid is *μ*, the shear stress *τ*_1_ is 2*μu*/*δ*. The range of shear stress is 0 to 800 Pa, and the range of the corresponding Reynolds number is 0 to 226. In shear flow, Ladd's momentum correction term [25] was used to solve the velocity boundary of the moving plates at the top and bottom of a fluid field:

(15) $$\begin{array}{c} f_{\bar{\alpha }}\left(x,t+∆t\right)=f_{\alpha }^{\left(\text{eq}\right)}\left(x,t\right)-\frac{2w_{\alpha }\rho }{c_{\text{s}}^{2}}\left(e_{\alpha }\cdot u\right), \end{array}$$

where $\bar{\alpha }$ is the opposite direction of *α*, **u**_*w*_ is the velocity of the boundary, and *c*_s_ is the Lattice velocity, which can be calculated from

(16) $$\begin{array}{c} c_{\text{s}}^{2}=c^{2}/3. \end{array}$$

The inlet and outlet were periodic boundary condition.

The blood cells will be impacted when flowing through the blood pump because of a high-speed rotating impeller. In impact flow, the RBC was impacted on the wall at certain velocity with fluid. The range of impact velocity is 0 to 10 m/s. Half-way bounce-back boundary was applied to solve the rebound of nodes of the membrane on the wall. Similar to shear flow, the inlet and outlet were periodic boundary condition.

The parameters of IB-LBM which is employed for solving the RBC in shear and impact flow are shown in Table 2.

## 3. Results and Discussion

### 3.1. The RBC in Shear Flow

The shapes of RBC stretched by different shear stresses are shown in Figure 2. The higher the shear stress is, the longer and narrower the RBC is, and the shape of RBC varies from biconcave to fusiform. The diameter of RBC in the long axis direction is about 13 *μ*m when the shear stress is 255 Pa. When the stress is 800 Pa, the diameter can be up to 17.5 *μ*m.

The change of RBC's free energy under different shear stresses is demonstrated in Figure 3. When the stress is larger than 150 Pa, the free energy increases obviously and has approximate linear relationship with shear stress. This case indicates that the membrane of RBC cannot resist the shear stress higher than 145 Pa. The hemolytic threshold value of RBC in shear flow is different according to past research. The most commonly used is 400 Pa [14]; others are 255 [13], 600 [7], and 800 Pa [5]; and the corresponding free energy added is 3.45 × 10^−14^, 2.04 × 10^−15^, 5.18 × 10^−15^, and 7.81 × 10^−15^ J, respectively, in this paper. The hemolytic threshold value of free energy is wide-ranging. In order to make sure of the hemolytic threshold value of free energy, other references and research are needed. The threshold free energy value of RBC's damage by impact was used in this paper.

Figure 4 illustrates the time needed for RBC's free energy to increase in different shear flow. The higher the shear stress is, the shorter the time spent is. When the shear stresses are 255 Pa, 400 Pa, 600 Pa, and 800 Pa, the corresponding time spent is 7.18 × 10^−1^, 6.51 × 10^−1^, 4.73 × 10^−1^, and 4.04 × 10^−1^ s, respectively.

As shown in Figure 5, the free energy increased over time when the RBC was shorn in 255, 400, 600, and 800 Pa shear flow. The tendency of free energy varying over time in different shear stresses was similar.

### 3.2. The RBC in Impact Flow

The biggest deformation of RBC in different impact flow is displayed in Figure 6. When the velocity of impact flow is 6, 8, and 10 m/s, the axial diameter of RBC in the long axial direction can be up to 14, 16, and 20 *μ*m, respectively. Not like the shape of RBC in shear flow, the deformation of RBC in impact flow seems to be compressed along the vertical direction of impact velocity.

The change of RBC's free energy, which comes to the biggest deformation in different impact velocities, is presented in Figure 7. As the impact velocity increases, the flatter RBC is squeezed and the free energy change is increased nearly linearly. When the velocity of impact flow is 10 m/s, the change of RBC's free energy is 4.135 × 10^−15^ J.

The processes of RBC's free energy changing in three kinds of impact velocity are demonstrated in Figure 8. The higher the impact velocity was, the bigger the increase of RBC's free energy was, and the time needed was shorter. Compared to Figure 5, the time needed in impact flow is much smaller than in shear flow, about an order of magnitude.

### 3.3. The RBC under Coupling Effect of Shear and Impact

Shear stress and high velocity simultaneously exist in the blood flow of the blood pump. The coupling effect of shear and impact should be analyzed. It is hard to simulate the RBC being shorn and impacted simultaneously. The parameters of nodes in the simulation of RBC being shorn were saved as the initialization state of impact flow in this paper for the simulation of the coupling effect of shear and impact. The free energy of RBC was changed significantly when shear stress was larger than 145 Pa according to Figure 3, so the range of shear stress between 145 and 400 Pa was selected in the simulation. Impact velocity varied from 0 to 8 m/s. The points in Figure 8 represented the simulation results of RBC's free energy in the coupling effect of different shear stresses and impact velocities. With the shear stress (*S*_s_) and impact velocity (*I*_v_) as variables, the values of RBC's free energy (*F*_e_) was fitted to be

(17) $$\begin{array}{c} F_{\text{e}}=1.02\sqrt{S_{s}^{2}+I_{v}^{2}}. \end{array}$$

*S*_s_ and *I*_v_ are the free energy of RBC changed with shear stress *x* (Pa) and impact velocity *y* (m/s), respectively, based on the data in Figures 3 and 7:

(18) $$\begin{array}{c} \left\{\begin{array}{c} S_{\text{s}}=0.012\left(x-145\right),\\ I_{\text{v}}=0.41y. \end{array}\right. \end{array}$$

The grid in Figure 9 is the result of Equation (16). The coupling effect of shear and impact was smaller than the addition of two effects, but larger than anyone alone.

## 4. Discussion

The RBC will be broken when the free energy of RBC is bigger than the threshold free energy of RBC for hemolysis. There are different threshold shear stresses for hemolysis in past researches for the different accuracy of research methods and expose time. In impact flow, the expose time is meaningless for the process of RBC being impacted must be complete. According to Yun and Tan [10], the threshold limit for hemolysis in impact flow is between 8 m/s and 10 m/s. According to fitting and interpolation of the data in Figures 3 and 7, when the RBC'S free energy change is the same, the impact velocity corresponding to the hemolytic threshold values of RBC in shear flow 255 Pa, 400 Pa, 600 Pa, and 800 Pa is 5.3 m/s, 8.68 m/s, 12.5 m/s, and 18.9 m/s, respectively. Because the impact velocity 8.68 m/s corresponding to the most commonly used hemolytic threshold value of RBC in shear stress 400 Pa is in this range, 8.68 m/s can be defined as the hemolytic threshold value of RBC in impact flow and the corresponding hemolytic threshold value of RBC's free energy *E*_0_ is 3.46 × 10^−15^ J.

In the research of Lu et al. [5], we know that when the shear stress is 800 Pa, the exposure time is 1 ms, and the RBC will be damaged. As shown in Figure 5, when the shear stress is 800 Pa, the exposure time is 2 ms, and the free energy can reach to *E*_0_. Therefore, the research is reasonable for the result of this paper comes close to the experiment result [5].

Equation (16) and *E*_0_ can be used for judgment of RBC being damaged in the coupling effect of shear and impact, and the RBC is damaged if the value of *F*_e_ is larger than *E*_0_.

## 5. Conclusions

Conclusions should clearly explain the main findings and implications of the work, highlighting its importance and relevance. The work of this paper can be summarized as follows:

1. The free energy, shape, and time needed for RBC when being shorn in different shear stresses are researched in the paper by using IB-LBM based on the WLC model
2. The free energy, shape, and time needed for RBC when being impacted in different impact flow were studied in the frame of the IB-LBM and WLC model
3. Combining the recent researches on the hemolytic threshold value of RBC in shear flow and impact flow with this paper's research on the changing of RBC's free energy when the RBC is shorn and impacted, we get the hemolytic threshold value of RBC's free energy which was about 3.46 × 10^−15^ J, the corresponding hemolytic threshold shear stress value of RBC is 400 Pa, and the impact velocity value of RBC is 8.68 m/s
4. An equation is built for judgment of RBC being damaged in the coupling effect of shear and impact based on the shear stress, impact velocity, and threshold value of RBC's free energy for hemolysis

The research of RBC's damage judgment is very important for the design and optimization of the blood pump. It is hard to judge the damage of RBC (hemolysis) in the blood pump in theoretical research, especially when the factors, which play a role on RBC, is not single, for example, the coupling effect of shear stress and impact. The research in this paper provides a way of judgment for RBC being damaged. Comparing the free energy of RBC in certain effects to the threshold free energy for hemolysis, if the free energy of RBC is larger, the RBC is damaged. The three-dimensional model will be applied in future work for more reasonable research on the mechanism of RBC being damaged.

## Figures and Tables

**Figure 1:** The simulation model of RBC in plasma. Two coordinate systems were used: Eulerian grid was used for the plasma and RBC cytoplasm, and Lagrangian grid was used for the RBC membrane. The RBC membrane was modeled as a series of particles (the number is 40) connected by a chain network which can resist compression/stretch and bending.

**Figure 2:** The shapes of RBC in different shear stresses (255 Pa, 400 Pa, 600 Pa, and 800 Pa) and the natural shape of RBC. The lager the shear stress was, the longer and narrower the RBC stretch was, and the shape of RBC varies from biconcave to fusiform.

**Figure 3:** Variation of RBC's free energy when the RBC is shorn in different shear stresses. The asterisk points present the data of computational result.

**Figure 4:** Variation of time needed for RBC's free energy to increase during RBC shearing in different shear stresses.

**Figure 5:** The RBC's free energy increased over time when the RBC was shorn in 255, 400, 600, and 800 Pa shear flow.

**Figure 6:** The shape of RBC when being impacted at different velocities.

**Figure 7:** Variation of RBC's free energy when the RBC is impacted in different velocities of flow.

**Figure 8:** The RBC's free energy changed over time when RBC is impacted in different velocities (6 m/s, 8 m/s, and 10 m/s) of flow.

**Figure 9:** The RBC's free energy changed in coupling effect of different shear and impact. The points represented the simulation result, and the grid represented the result of fitted equation.

**Table 1:** Parameters of the RBC model and IB-LBM.

Parameter	Value	LBM value
*k*_L_	5.22 × 10^−18^ nm	1.8 × 10^−5^
*k*_B_	5.80 × 10^−18^ nm	2.0 × 10^−6^
*k*_S_	5.22 × 10^−15^ nm	1.8 × 10^−2^
Plasma density *ρ*	1.0 g/cm^3^	1
Plasma kinetic viscosity *μ*_*ρ*_	1.2 × 10^−6^ m^2^/s	0.01
Reference area *s*_0_	27.7 *μ*m^2^	690

**Table 2:** The parameters of IB-LBM.

Parameter	Value	IB-LBM value
Space size	1 *μ*m	5
Time step Δ*t*	3 × 10^−8^ s	1
Lattice unit *δ*_*x*_		1
Lattice unit *δ*_*y*_		1
Lattice velocity *c*_s_		3^-1/2^

## Data Availability

The simulation result of RBC being stretched for verification of the RBC model is available at 10.3938/jkps.74.607 and is cited at relevant places within the text as [20]. The threshold limit of shear stress for hemolysis is available at 10.1016/S0021-9290(01)00084-7, 10.1007/s10237-005-0005-y, 10.1002/fld.3939, and 10.1016/j.mvr.2011.05.006 and is cited at relevant places within the text as [5, 7, 13, 14], respectively. The free energy of RBC in different shear stress, impact velocity, and coupling effects of shear and impact which is used to support the findings of this study is available from the corresponding author upon request.
